This article has been retracted.

# Metabolic Differences between Ex-Smokers and Nonsmokers: A Metabolomic Analysis

**DOI:** 10.1155/2022/6480749

**Published:** 2022-04-16

**Authors:** Lirong Liang, Lin Feng, Long Zhou, Shuilian Chu, Di Zhang, Hang Jin, Jiachen Li, Liancheng Zhao, Zhaohui Tong

**Affiliations:** ^1^Department of Research on Tobacco Dependence Therapies Beijing Institute of Respiratory Medicine and Beijing Chao-Yang Hospital, Capital Medical University, Beijing, China; ^2^Department of Cardiology Sichuan Provincial People's Hospital, University of Electronic Science and Technology of China, Chengdu, China; ^3^Division of Prevention and Community Health National Center for Cardiovascular Disease Fuwai Hospital, Chinese Academy of Medical Sciences and Peking Union Medical College, Beijing, China; ^4^Department of Respiratory and Critical Care Medicine Beijing Institute of Respiratory Medicine and Beijing Chao Yang Hospital, Capital Medical University, Beijing, China

## Abstract

The aim of this study was to compare changes in the metabolite levels of ex-smokers and nonsmokers using a metabolomics approach, accounting for the weight gain in ex-smokers. Volunteer ex-smokers and nonsmokers were recruited from two cohorts Shijingshan (174) and Xishan (78), respectively, at a 1 : 1 ratio for age and sex. Nontargeted metabolomics was performed on the volunteers' blood samples using liquid chromatography-mass spectrometry, and multivariate statistical analysis was performed using principal component analysis and orthogonal partial least squares discriminant analysis. Enrichment analysis was used to identify Kyoto Encyclopedia of Genes and Genomes (KEGG) pathways associated with differential metabolites and weighted gene co-expression network analysis and maximal correlation coefficient (MCC) algorithms were used to identify key metabolites. The results revealed no significant differences between the distribution of blood metabolite levels in the ex-smokers and nonsmokers. The biosynthesis of valine, leucine, and isoleucine was determined to be associated with differential metabolites, and five key metabolites were identified. Further analysis revealed differences in weight gain and regained metabolite levels in ex-smokers, and 10 differential metabolites were identified that may be associated with weight gain in ex-smokers. These findings suggest that quitting smoking restores metabolites to almost normal levels and results in weight gain. The identified key metabolites and metabolic pathways may also provide a basis for clinical studies.

## 1. Introduction

Tobacco use is a major risk factor for disability and premature death, and it imposes a global burden of disease [1]. In 2019, about 114 million people worldwide were smokers, consuming about 7.41 trillion equivalents of tobacco [2]. The distribution of smokers shows regional differences. The 2015 Global Burden of Disease Study estimated that the prevalence of smoking was significantly higher in Europe and Southeast Asia than the global prevalence, while the lowest prevalence was found in western sub-Saharan Africa.

Smoking-related diseases are a significant burden on global public health, and smoking accounts for an average of five million lives per year [3]. In 2019, there were 200 million and 769 million disabilities and deaths due to smoking, respectively. The risk of disease in the smoking population is significantly higher than in the nonsmoking population. Smoking is a major cause of lung disease, it accelerates the disease process in patients with asthma, and it is a significant risk factor for chronic obstructive pulmonary disease and lung cancer [4]. In addition, smoking induces the development and progression of diseases, including gastrointestinal diseases [5], cardiovascular diseases [6], and cancer [7]. The occurrence of these diseases often imposes a great burden on families and society. In the case of lung cancer, for example, the risk of developing lung cancer is about 20 times higher in smokers than in nonsmokers [7]. On an economic level, nonsmokers incur about half the cost of disease treatment compared to smokers [8].

Due to the excessive disease burden, a large number of smokers are deciding to cease smoking. However, it has been found that compared to nonsmokers, previously heavy smokers have a significantly increased risk of disease five years after quitting [8]. Other studies have shown that this increased risk may be associated with genome-wide alterations [9]. Moreover, smoking cessation is often accompanied by weight gain [1, 10–12]. In general, weight gain is associated with increased risk of major chronic diseases and decreased odds of healthy living. Therefore, smoking cessation related weight gain may reduce the health benefits of quitting smoking [13–15]. However, the underlying mechanism of weight gain after quitting is not fully clear.

Recently, the relationship between the metabolome and disease has attracted attention. The metabolome is the product of gene expression in an organism and is present in cells, tissues, organs, or organisms. The metabolome constitutes a vast network of metabolic reactions, and the differences between the metabolites of patients and normal subjects can be analyzed to identify disease biomarkers and develop diagnostic methods. Hence, in this study, we aimed to compare the metabolites of ex-smokers with those of nonsmokers and to identify the possible metabolic pathways contributing to any differences and exploring the potential metabolome-related mechanism of weight gain after quitting.

## 2. Materials and Methods

### 2.1. Data Sources

The volunteer participants were first divided into two cohorts (Shijingshan and Xishan), and then into two groups, ex-smokers and nonsmokers matched 1 : 1 according to age and sex within each cohort. The Shijingshan cohort contained 87 ex-smokers and 87 nonsmokers, and the baseline survey was conducted in 2010 and the resurvey was conducted in 2015. The Xishan Gun Factory cohort contained 39 ex-smokers and 39 nonsmokers and was first surveyed at in 2007 and resurveyed in 2012. The participants were defined as the nonsmokers who were never smokers at the two surveys with the 5-year interval and were defined as the ex-smokers who were former smokers at the two surveys. The participants' age range was 35–75 years old, and they did not have cardiovascular diseases, stroke, lung, or liver disease. In addition, the weight gain was defined as the 5-year difference of weight ≥2 kg measured at the resurvey subtracted by the weight measured at the first survey. Blood samples were collected separately, and plasma samples were obtained by centrifugation and stored at −70°C.

### 2.2. Nontargeted Metabolomics Analysis

The plasma samples were pretreated and the supernatant was obtained by a protein precipitation method. The supernatant was analyzed using liquid chromatography (HPLC). A SCIEX, UK liquid phase system was used for data acquisition, and the column used was an ACQUITY UPLC T3 (100 mm ∗ 2.1 mm, 1.8 *μ*m, Waters, UK). The column temperature was set at 35°C and the flow rate was 0.4 ml/min. The mobile phases used were phase A: water (0.1% formic acid) and phase B: acetonitrile (0.1% formic acid). It was translated with https://www.DeepL.com/Translator (free version).

### 2.3. Principal Component Analysis (PCA)

The ex-smoker groups were used as the test groups, and the nonsmoker groups were used as the control groups. The metabolite levels of the test and control groups were compared. Multivariate statistical analysis was performed using principal component analysis (PCA) and orthogonal partial least squares discriminant analysis (OPLS-DA) on all the metabolic characteristics of the test groups. PCA was mainly used to visualize differences in distribution between the ex-smoker and nonsmoker groups, and OPLS-DA was mainly used to select differential metabolic characteristic ions that distinguished the two groups.

### 2.4. Metabolite Identification

The metabolic phenotypes of the ex-smoker and nonsmoker groups were assessed using KEGG pathway enrichment analysis to observe the differences between the metabolite levels of the two groups. Pathway enrichment analysis was performed using all metabolic signatures with a threshold of *P* < 0.05. Metabolite identification and annotation were based on HPLC and used reliable in-house and online databases.

### 2.5. Selection of Key Metabolites

After excluding samples that lacked clinical phenotypes from the Shijingshan cohort, the metabolite profiles of 166 samples were included in a weighted gene co-expression network analysis (WGCNA), and *β* = 22 was selected as a soft threshold for network development. Co-expression modules were identified and their characteristics were analyzed. The adjacency matrix was transformed into a topological overlap matrix network to build gene dendrograms and module colors. Hierarchical clustering of modules was performed by calculating the differences in module Eigen objects and merging similar modules. The metabolite-metabolite module-phenotype (body mass index [BMI], etc.) axes were constructed to resolve the metabolite changes and biological process differences found in the ex-smoker groups. The correlation between modules and phenotypes was calculated using the Pearson method, and the modules with the highest correlation were selected to identify the top five key metabolites using the MCC plug-in of Cytoscape software and to analyze the metabolite-related pathways.

## 3. Results

### 3.1. Unsupervised Learning Methods: PCA

The multivariate statistical methods PCA and OPLS-DA were used to analyze the nonsmoker and ex-smoker groups of the Shijingshan cohort. The results are shown in Figure 1. Ex-smoker and nonsmoker samples could be distinguished by the model; however, the difference was less significant. This indicates that the metabolite levels of the ex-smokers were similar to those of the nonsmokers. However, a small portion of the sample were outliers, indicating that there was heterogeneity in the population, and that some of the ex-smokers had metabolic profiles that were different from those of the other ex-smokers and the nonsmokers. In addition, the S-plot multivariate data processing technique could discriminate potential markers in the model, and markers with VIP values greater than 2.0 were considered potential markers.

We then analyzed the relationship between smoking cessation and weight gain in the Xishan cohort. As shown in Figures 2(a) and 2(b), the difference between the distribution of those who gained weight and those who did not gain weight in the ex-smoker group was more pronounced, and the difference was more significant in the 2012 data than in the 2007 data. This indicates that there may be some weight gain after quitting smoking. We then focused on the intersection of the differential metabolites of these two data sets to identify 10 common metabolites.

### 3.2. KEGG

Based on the 174 Shijingshan cohort samples used for metabolite detection analysis, 93 differential metabolites were identified and used for KEGG pathway analysis. As seen in Table 1, the differential metabolites were mainly related to the synthesis and degradation of amino acids or proteins, with the most significant pathways being the biosynthesis of valine, leucine, and isoleucine.  Figure 3 illustrates this finding and depicts the biosynthesis of valine, leucine, and isoleucine using pathway maps.

### 3.3. WGCNA

With phenotypes (cohort genus, smoking cessation status, BMI, etc.) used as feature profiles and metabolic profiles used as network construction objects, the metabolic profiles were analyzed for weighted metabolite co-expression regulatory networks using the WGCNA algorithm. All metabolites were divided into five color modules (Figure 4(a)), and the clustering diagrams depicting the relationships between them are shown in Figure 4(b). The strongest correlation between the analyzed modules and phenotypes was between the GREY module and phenotypes, such as smoking cessation status and BMI (Figure 4(c)). The metabolites included in this color module are shown by the circle diagram (Figure 4(c)). The five most significant metabolites were Nb-palmitoyl tryptamine, palmitic acid, ganolucidic acid C, hovenidulcigenin A, and argenteane (Figure 4(e)).

## 4. Discussion

Metabolomics is used to comprehensively analyze metabolites to provide a systematic view of the biological processes of diseases. It supports disease diagnosis, pathogenesis, and interventions by detecting potential biomarkers and metabolic pathways [16]. In this study, we performed a metabolomic analysis of ex-smokers and nonsmokers using HPLC and determined KEGG pathways associated with differential metabolites through multivariate statistical analysis of the metabolites found in the ex-smoker and nonsmoker groups. In addition, the effects of smoking cessation on weight gain and meaningful metabolites were determined.

The multivariate statistical analysis showed that the difference in metabolite levels between the ex-smoker group and the nonsmoker group was not significant, reflecting that metabolic levels may return to normal levels after five-year smoking cessation.

This study also examined the effect of smoking cessation on body weight by analyzing body weight changes in ex-smokers of Xishan cohort from 2007 to 2012. It was found that there was a more significant difference in the data distribution between the weight-gain group and the non-weight-gain group after quitting. The relationship between smoking cessation and weight gain was reported in the last century [17]; those who successfully quit smoking experienced a significant increase in BMI three months after the first examination [18].

Based on this information, we used WGCNA to identify metabolites associated with both smoking status and BMI changes in phenotypes in the Shijingshan cohort. The five most relevant metabolites were Nb-palmitoyl tryptamine, palmitic acid, ganolucidic acid C, hovenidulcigenin A, and argenteane. Palmitic acid is a saturated fatty acid, and an elevated blood concentration leads to an inflammatory response [19]. The remaining metabolites are less studied. The differential metabolites of the weight-gain and non-weight-gain groups of the Xishan cohort (2007 and 2012) were also examined, and 10 common metabolic profiles were identified.

The metabolic pathways affected by lifestyle behaviors can be understood by detecting changes in blood metabolites of ex-smokers and nonsmokers. Based on this conclusion, we performed a KEGG pathway enrichment analysis of differential metabolites in the Shijingshan cohort, and the results pointed to a unique pathway: the biosynthesis of valine, leucine, and isoleucine. Leucine increases protein synthesis, stimulates insulin release, and is an important metabolic signal in skeletal muscle [20]. Isoleucine is associated with liver and fat metabolism and can facilitate energy metabolic processes [21]. Valine, leucine, and isoleucine are all branched-chain amino acids (BCAAs). In contrast to the role of individual BCAAs, when combined, the three amino acids regulate lipid metabolism and fat deposition and are signaling pathways for protein synthesis, glucose homeostasis, anti-obesity activity, and nutrient sensitivity [22, 23]. However, BCAAs have also been associated with a variety of diseases; their metabolism can influence a variety of disease phenotypes and they can act as biomarkers during disease progression [24, 25]. It has been shown that smoking has an interactive effect on plasma uric acid and plasma-free amino acid levels. Smokers have significantly lower serum concentrations of BCAAs, with an increased risk of worsening lung function [26].

Currently, there is an increasing interest in using metabolomic analysis to study smoking-related diseases; however, there are few studies on the effect of smoking cessation on metabolites. Here, we analyzed the metabolites of ex-smokers and nonsmokers from a metabolomics perspective using HPLC techniques and multivariate statistical analysis and concluded that metabolite levels generally return to normal after smoking cessation. The KEGG pathway associated with the differential metabolites was identified using enrichment analysis. Five key metabolites were identified using the WGCNA and MCC algorithms. It was also concluded that there were differences in weight gain in the ex-smoker population, which will be needed to elucidate the mechanism underlying weight gain after smoking cessation in the future.

## Figures and Tables

**Figure 1:** Score plots for the Shijingshan cohort's ex-smoker and nonsmoker groups. (a) PCA score plots of metabolite content in ex-smoker versus nonsmoker samples in positive and negative ion mode; (b) OPLS-DA score plots of metabolite content in ex-smoker versus nonsmoker samples in positive and negative ion mode; and (c) S-plot of the model in positive and negative ion mode.

**Figure 2:** The metabolite scores for weight gain in the Xishan cohort's ex-smoker and nonsmoker groups. (a) OPLS-DA score plot of the 2007 survey weight gain data with and without positive ions and negative ions model; (b) OPLS-DA score plot of the 2012 survey weight gain data with and without positive ions and negative ions model; and (c) intersection of the differential metabolites for weight gain with and without a group using the 2007 and 2012 ex-smoker groups.

**Figure 3:** Construction of KEGG-related metabolic pathways. (a) Pathways related to metabolites and (b) pathway maps of valine, leucine, and isoleucine biosynthesis.

**Figure 4:** The WGCNA used to identify the key metabolites. (a) Clustering diagram of WGCNA screening modules and metabolites; (b) clustering diagram showing the relationships between the modules; (c) correlation heat map of each phenotype and each module; (d) linkage relationship circle diagram of key modules; (e) top five key metabolites.

**Table 1:** KEGG pathway analysis results.

Pathway	Total	Expected	Hits	Raw p	Holm p	FDR	Impact
Valine, leucine, and isoleucine biosynthesis	8	0.14452	2	0.0082418	0.69231	0.69231	0
Biosynthesis of unsaturated fatty acids	36	0.65032	2	0.13613	1	1	0
Valine, leucine, and isoleucine degradation	40	0.72258	2	0.16139	1	1	0.01084
Phenylalanine metabolism	10	0.18065	1	0.16709	1	1	0
Aminoacyl-tRNA biosynthesis	48	0.8671	2	0.21414	1	1	0
Pantothenate and CoA biosynthesis	19	0.34323	1	0.29419	1	1	0
Ether lipid metabolism	20	0.36129	1	0.3071	1	1	0.14458
Sphingolipid metabolism	21	0.37935	1	0.31978	1	1	0.02434
Glycerophospholipid metabolism	36	0.65032	1	0.48514	1	1	0.01736
Fatty acid elongation	39	0.70452	1	0.5132	1	1	0
Fatty acid degradation	39	0.70452	1	0.5132	1	1	0
Tryptophan metabolism	41	0.74065	1	0.53108	1	1	0.14305
Primary bile acid biosynthesis	46	0.83097	1	0.57305	1	1	0
Fatty acid biosynthesis	47	0.84903	1	0.581	1	1	0.01473

Total is the number of all metabolites in this metabolic pathway; hits is the number of differential metabolites in this metabolic pathway screened in this study; raw *p* indicates the originally calculated *P* value for the enrichment analysis; Holm *p* indicates the *P* value for the Holm–Bonferroni statistical method used in the enrichment analysis; and FDR *p* indicates the FDR error control *P* value for the multiplex test, and impact is the metabolic pathway impact value. A *P* < 0.05 was considered statistically significant.

## Data Availability

The datasets used and analyzed during the current study are available from the corresponding author on reasonable request.
